The article "An Extract of Antrodia camphorata Mycelia Attenuates the Progression of Nephritis in Systemic Lupus Erythematosus-Prone NZB/W F1 Mice" was published in 2011. Journal: Evid Based Complement Alternat Med.

# An Extract of *Antrodia camphorata* Mycelia Attenuates the Progression of Nephritis in Systemic Lupus Erythematosus-Prone NZB/W F1 Mice

**DOI:** 10.1093/ecam/nen057

**Published:** 2011-02-17

**Authors:** Jia-Ming Chang, Yi-Ru Lee, Le-Mei Hung, Sheng-Yung Liu, Mao-Tien Kuo, Wu-Che Wen, Peini Chen

**Affiliations:** ^1^Division of Research and Development, Development Center for Biotechnology, Xizhi City, Taipei County, Taiwan 221, Taiwan; ^2^Institute of Molecular Biology and Biochemistry, College of Medicine, National Taiwan University, Taiwan 111, Taiwan; ^3^Golden Biotechnology Corp., Danshuei Township, Taipei County, Taiwan 251, Taiwan; ^4^Department of Radiology, Taipei Veterans General Hospital, Taipei, Taiwan 112, Taiwan

## Abstract

*Antrodia camphorata* is used in folk medicine for the treatment of inflammation syndromes and liver-related diseases in Taiwan. The goal of this study was to evaluate the efficacy of the mycelial extract of *A. camphorata* (ACE) for the treatment of systemic lupus erythematosus (SLE) in SLE-prone NZB/W F1 mice. After antibodies against double-stranded DNA appeared in NZB/W mice, the mice were orally administered varying dosages of ACE (100, 200 and 400 mg kg^−1^) for 5 consecutive days per week for 12 weeks via gavage. To assess the efficacy of ACE, we measured SLE-associated biochemical and histopathological biomarkers levels of blood urine nitrogen (BUN), blood creatinine, urine protein and urine creatinine and thickness of the kidney glomerular basement membrane by staining with periodic acid-Schiff. Antroquinonol, an active component of ACE, was investigated for anti-inflammation activity in lipopolysaccharide-induced RAW 267.4 cells. ACE at 400 mg kg^−1^ significantly suppressed urine protein and serum BUN levels and decreased the thickness of the kidney glomerular basement membrane. Antroquinonol significantly inhibited the production of tumor necrosis factor-**α** and interleukin-1**β** by 75 and 78%, respectively. In conclusion, ACE reduced urine protein and creatinine levels and suppressed the thickening of the kidney glomerular basement membrane, suggesting that ACE protects the kidney from immunological damage resulting from autoimmune disease.

## 1. Introduction

Systemic lupus erythematosus (SLE) is an autoimmune disease for which the pathogenesis remains unclear [1]. Patients with SLE produce numerous antibodies against self-antigens in several organs, such as skin, joints and kidneys [2]. The clinical features include fever, photosensitivity, serositis [3] and renal disease, the latter being the most life threatening due to potential development of irreversible kidney failure [4].

It has been suggested that in SLE hyperactive B cells produce auto-antibodies against DNA fragments. These antibodies can then attack the nuclear antigens of organs or form immunocomplex precipitates that affect microcirculation, resulting in organ dysfunction [2]. When precipitated immunocomplexes in the kidney result in glomerulitis, patients will present with significant amounts of protein in the urine. Furthermore, the thickness of glomerular basement membranes is increased in glomerulitis and results in the reduction of blood creatinine clearance, which serves as an important diagnostic parameter for lupus nephritis [5].

The BXSB, MRL/lpr and NZB/W F1 mouse models have been commonly used to validate drug regimens for the treatment of SLE. Male BXSB mice characteristically develop SLE faster than females, which is opposite of that observed in humans [6]. MRL/lpr mice are characterized by lymphadenosis, splenomegaly and polyarthritis. In NZB/W F1 mice, females spontaneously produce auto-antibodies at 5-6 months of age and the mice die from kidney failure. Among these mouse models, the symptoms of SLE-prone NZB/W F1 mice are most similar to those of human SLE patients [7, 8] and therefore provide the most promising model for evaluation of anti-SLE drug activity.

*Antrodia camphorata* (Polyporaceae, Aphyllophorales), a parasitic fungus on rotting trees of *Cinnamomum kanehirai* Hay [9], is used in Taiwanese folk medicine for the treatment of diarrhea, abdominal pain, hypertension, itching of the skin and liver cancer. To date, *A. camphorata* has been cultured as mycelium and has been shown to exhibit certain anti-inflammation [10, 11], vasorelaxation [12] and anti-tumor cytotoxicity [13, 14] activities. However, the ability of *A. camphorata* to inhibit auto-immune diseases has not been subjected to scientific scrutiny.

To assess the anti-SLE efficacy of *A. camphorata* mycelia, we treated SLE-prone NZB/W F1 mice with extracts of a *camphorata* mycelia and measured the diagnostic parameters associated with lupus nephritis. Furthermore, RAW 264.7 cells, a mouse leukemic monocyte macrophage cell line, were treated with the active ingredient of the extract, antroquinonol, to evaluate its anti-inflammation activity.

## 2. Methods

### 2.1. Cells and Chemicals

RAW 264.7 cells (TIB-71) were obtained from the American Type Culture Collection (Manassas, VA, USA). ACE and antroquinonol were provided by Golden Biotechnology Co. (Taiwan). Prednisolone was used as a positive control and was purchased from Chin Teng Pharmacy Industrial Co. (Taiwan). Lipopolysaccharide (LPS) was purchased from Sigma Co. (USA). All drugs were stored at −20°C and thawed at 37°C before use.

### 2.2. Animals

Fifty NZB/W F1 female mice were purchased from Jackson Laboratory (Bar Harbor, ME, USA) and mice were maintained under climate-controlled conditions and a 12 hours light-dark cycle. The animals were fed standard rodent chow (PMI Nutrition International, USA). Ten C57BL/6j female mice were purchased from the Animal Center of the National Taiwan University and were used as reference controls. All mice received human care and the study protocol followed the guidelines of the Institutional Animal Care and Use Committees of the Development Center for Biotechnology (accredited by AAALAC).

### 2.3. Preparation of ACE

The *A. camphorata* used in this study was authenticated by Dr Tzean Shang-Shong, Department of Plant Pathology and Microbiology, National Taiwan University, Taiwan. The mycelium of *A. camphorata* was cultured in 1000 mL growth medium containing 0.1 g NaCl, 10 g peptone, 2 g yeast extract, 10 g agar and 10 g cereal mixture (rice, wheat or corn), pH 7.5 at 25°C for 12–14 weeks. After cultivation, 500 g of lyophilized *A. camphorata* mycelium was extracted with 2500 mL *n*-hexane for 6 hours. The *n*-hexane fraction, defined as ACE (GD-66, product name and GD-AIDT7, batch name), was concentrated to 20–30 mL via vacuum evaporation and the antroquinonol was purified from ACE by silica gel chromatography (column = 45 cm, 5 cm i.d.) (ASTM silica gel, Merck Co., Germany) and eluted with *n*-hexane : ethyl acetate (10 : 3 v/v). The resulting eluate was further subjected to size exclusion chromatography using Sephadex LH20 column (70 cm long, 5 cm i.d.) (AB gel, GE Healthcare Bio-Science, USA). The antroquinonol (98% purity) was eluted with 95% ethanol as described in the study of Lee et al. [9]; the ACE fraction was determined to have 0.01% antroquinonol.

### 2.4. Drug Treatment

After NZB/W F1 mice were 23 weeks old, blood was collected for determination of IgG against double-stranded DNA (anti-dsDNA). Mice positive for anti-dsDNA IgG were divided into five groups of 10 mice each and treated with various concentrations of ACE or prednisolone by gavage for 5 consecutive days per week for 12 weeks as follows: (i) disease group, ddH_2_O treatment (10 mL kg^−1^), (ii) positive control group, prednisolone treatment (1.25 mg kg^−1^), (iii) ACE treatment (100 mg kg^−1^), (iv) ACE treatment (200 mg kg^−1^) and (v) ACE treatment (400 mg kg^−1^) (Table 1). Ten C57BL/6j mice were used as reference group in this experiment.

### 2.5. Analysis of Blood Urea Nitrogen and Urine Protein

For analysis of blood urea nitrogen (BUN), serum samples were thawed at room temperature and then loaded on a BUN diagnostic kit slide. BUN was measured using an automated analyzer (BUN_Vitros DT6011, Johnson-Johnson, USA). For analysis of urine protein, urine was collected by pressing the bladder of mice with fingertips every 2 weeks. Urine protein was determined using the Bio-Rad Protein Assay Dye Reagent Concentrate according to the manufacturer's instructions, using bovine serum albumin as the standard. Optical density (OD) was measured at 595 nm.

### 2.6. Analysis of Serum and Urine Creatinine

Creatinine was determined by a Creatinine (Direct) Reagent Set (Eagle Diagnostics), according to the manufacturer's instruction. The urine samples were diluted with deionized water (1 : 10) and mixed with an equal volume of the diluted reagent provided in the kit in a 96-well microtiter plate and incubated for 15 min at room temperature. The OD at 510 nm was then determined and the concentration of urine creatinine was calculated as follows: creatinine (mg dL^−1^) = [(sample OD-blank OD) × 6 mg dL^−1^/(sample OD-blank OD)]. Serum creatinine was measured using the urine creatinine protocol but no dilution was needed for measuring serum creatinine.

### 2.7. Determination of Serum Anti-dsDNA IgG

The levels of anti-dsDNA IgG were determined using a mouse anti-dsDNA IgG ELISA kit (Alpha Diagnostic, USA), according to the manufacturer's instructions. In brief, blood serum samples were diluted 100-fold with buffer (provided by the kit) and added to a 96-well ELISA plate and incubated for 2 hours at room temperature. Samples were then washed thrice with washing buffer (provided by the kit) and horseradish peroxidase–conjugated anti-IgG antibodies were then added and incubated for 1 hour at room temperature. The samples were washed five times with washing buffer and horseradish peroxidase substrate solution was added and incubated for 15 min at room temperature. The OD was measured at 450 nm using an ELISA reader. (Multiskan EX, Thermo Scientific Co., USA). The concentration of the anti-dsDNA was calculated using a bovine serum albumin standard calibration curve.

### 2.8. Histopathological Examination

After sacrificing the animals, the kidneys were collected. A pathological examination was performed and sections were paraffin fixed and stained by haematoxylin and eosin and periodic acid-Schiff (PAS). PAS was used to stain the kidney glomerular basement membrane.

### 2.9. Anti-Inflammation Assay

RAW 264.7 cells were seeded onto a 24-well plate at a density of 5 × 10^5^ cells/well and incubated at 37°C for 24 hours under 5% CO_2_. RAW 264.7 cells were treated with varying concentrations of antroquinonol (MW 391) (0.256, 2.56, 25.6 and 256 *μ*M) for 24 hours in the presence of 1 *μ*g mL^−1^ LPS. After treatment, the medium was analyzed by ELISA to determine the secretion of tumor necrosis factor-*α* (TNF-*α*) and interleukin (IL)-1*β* cytokines, as described in the study of Chang et al. [15].

### 2.10. Statistical Analysis

Statistical analysis of *in vivo* data was performed using one-way ANOVA (SPSS software package). *In vitro* data were analyzed using the Student's *t*-test. Differences in values were considered significant at *P* < .05.

## 3. Results

### 3.1. Decreased Serum BUN Levels in ACE-Treated NZB/W Mice

Fifty NZB/W F1 female mice were divided into 5 groups of 10 mice each. Varying doses of ACE and prednisolone were administrated by gavage 5 consecutive days/week for 12 weeks. The body weight of NZB/W F1 mice was recorded every 2 weeks (Table 2). The growth of NZB/W F1 mice was not affected in the ACE- and prednisolone-treated groups, whereas the growth was significantly inhibited (only a 1.1% increase in body weight compared to initial body weight) in vehicle-treated NZB/W F1 mice at the end of the 12 week experiment. Mice displayed an increase in body weight of 3.1, 6.0 and 6.5%, when treated with 100, 200 and 400 mg kg^−1^ doses of ACE, respectively. The increase in body weight reflected the improved condition of SLE mice, suggesting that ACE might improve the cachexia symptoms of SLE disease.

To evaluate whether kidney function in SLE-prone NZB/W F1 mice was protected by ACE, serum creatinine and BUN levels were analyzed following the 12 week ACE treatment regimen. As shown in Figure 1(a), BUN levels were elevated to 49.5 ± 1.0 mg dL^−1^ in vehicle-treated NZB/W F1 mice, whereas BUN levels were decreased to 14.2 ± 0.6 mg dL^−1^ in prednisolone-treated mice. Likewise, BUN levels were decreased among mice treated with different doses of ACE (23.0 ± 9.7 mg dL^−1^ for 100 mg kg^−1^ ACE group, 17.8 ± 3.5 mg dL^−1^ for 200 mg kg^−1^ ACE group and 17.8 ± 3.3 mg dL^−1^ for 400 mg kg^−1^ ACE group). Thus, at dosages of 200 and 400 mg kg^−1^, ACE treatment decreased BUN levels by 64%. Furthermore, lower creatinine levels were observed in the prednisolone group (0.67 mg dL^−1^) and ACE groups (0.69 mg dL^−1^ in 100 mg kg^−1^ treatment group and 0.62 mg dL^−1^ in 400 mg kg^−1^ treatment group) compared to SLE-disease group (0.81 mg dL^−1^) (Figure 1(b)). Furthermore, prednisolone treatment decreased serum creatinine levels to 0.67 ± 0.05 mg dL^−1^ in NZB/W F1 mice as did ACE treatment (serum creatinine = 0.69 ± 0.10 mg dL^−1^ in the 100 mg kg^−1^ ACE treatment group and 0.62 ± 0.07 mg dL^−1^ in the 400 mg kg^−1^ ACE treatment group) compared to SLE-disease group of NZB/W F1 mice (serum creatinine = 0.81 ± 0.14 mg dL^−1^). These results suggested that kidney function, including serum creatinine clearance, is maintained by ACE treatment. 

### 3.2. Attenuation of Nephritis in SLE-Prone NZB/W F1 Mice

To evaluate the severity of nephritis in ACE-treated NZB/W F1 mice, urine protein and creatinine were analyzed, which are indicators of severity for lupus nephritis. The concentration of urine protein in the SLE disease group was dramatically increased to 581.8 ± 298.7 mg dL^−1^ at the end of the 12 week experiment, which was consistent with the body weight loss and indicated the onset of nephritis (Figure 1(c)). Prednisolone inhibited the increase in the levels of urine protein by 82% and 100, 200 and 400 mg kg^−1^ per dose of ACE inhibited urine protein by 69, 62 and 55%, respectively. As shown in Figure 1(d), the levels of urine creatinine were normal in the SLE-disease group (40.9 ± 0.6 mg dL^−1^) but were increased in prednisolone-treated mice (53.4 ± 5.1 mg dL^−1^). In contrast, mice treated with 400 mg kg^−1^ per dose of ACE had decreased urine creatinine (34% lower) compared to the SLE-disease group. Compared to creatinine in the blood, ACE maintained the glomerular function of kidneys in clearance of creatinine.

### 3.3. ACE Modestly Decreases the Production of Serum Anti-dsDNA Antibodies

In SLE, the levels of serum anti-dsDNA increase with the progression of SLE. As shown in Figure 2, the levels of anti-dsDNA IgG in vehicle-treated NZB/W F1 mice were dramatically elevated to 145.8 ± 46.4 mg dL^−1^ at the end of the 12 week period compared to the reference normal C57BL/6j mice (1.72 ± 0.05 mg dL^−1^), suggesting that SLE was successfully established. Unexpectedly, the levels of anti-dsDNA IgG were not inhibited by prednisolone (144.5 ± 95.8 mg dL^−1^) but the levels of anti-dsDNA IgG were reduced to 79.6 ± 18.7 mg dL^−1^ (45% inhibition) and to 123.9 ± 27.6 mg dL^−1^ (15% inhibition) in NZB/W F1 mice treated with 100 and 200 mg kg^−1^ per dose of ACE, respectively. Treatment of mice with 100 mg kg^−1^ per dose of ACE reduced the production of auto-antibodies, suggesting that the suppression of the immune response might be one of the pharmaceutical actions of ACE.

### 3.4. ACE Treatment Protects Kidneys via Inhibition of Glomerular Basement Membrane Thickening

Because death among SLE patients typically results from nephritis, we examined the capillary walls of the kidney glomeruli by staining with PAS. As shown in Figure 3, prednisolone suppressed thickening of the glomeruli basement membrane to 11 ± 1.32 *μ*m in SLE-prone mice, whereas the thickness of the glomeruli basement membrane was 23 ± 2.98 *μ*m in vehicle-treated mice. Thickening of the kidney glomeruli basement membrane was also significantly suppressed by ACE treatment in a dose-dependent manner (thickness = 19.1 ± 2.6 *μ*m, 17.5 ± 2.6 *μ*m and 17 ± 1.7 *μ*m for mice treated with 100, 200 and 400 mg kg^−1^ per dose of ACE, respectively. Although ACE treatment only moderately inhibited thickening of glomerular basement membrane, it did protect the kidney glomeruli from immunological damage. These results suggested that ACE treatment attenuated the onset of nephritis, thereby reducing the risk of death.

### 3.5. Anti-Inflammation of Antroquinonol

To understand the possible mechanism of ACE action, antroquinonol, the major component of ACE, was investigated for anti-inflammatory activity. RAW 264.7 cells were treated with antroquinonol at 0.256, 2.56, 25.6 and 256 *μ*M. Antroquinonol inhibited the production of TNF-*α* and IL-1*β* in LPS-induced inflammation in a dose-dependent manner (Figures 4(a) and 4(b)). In particular, a dose of 256 *μ*M antroquinonol inhibited LPS-induced TNF-*α* and IL-1*β* secretion by 75 and 78%, respectively. This result showed that antroquinonol might exert anti-inflammation activities in ACE-treated SLE-prone mice.

## 4. Discussion

Nephritis in SLE patients is the major cause of death due to auto-immune destruction of the kidneys. Elevated urine protein and BUN are also observed among patients with nephritis [16]. In this study, an extract of a *camphorata*, a herbal medicine used in Taiwan, maintained normal growth among SLE-prone mice and protected the kidneys from immunological damage, allowing for normal kidney function with respect to clearance of BUN and creatinine. Additionally, the thickening of the kidney glomerular basement membrane was suppressed, suggesting that ACE attenuated the progression of nephritis in SLE-prone mice. Taken together, these results demonstrate that ACE protects kidney function in SLE-prone animals via an unknown mechanism, suggesting that ACE may have efficacy for treatment of SLE.

Pro-inflammatory cytokines play a central role in acute and chronic liver inflammation. Among these pro-inflammatory cytokines, TNF-*α* and IL-1*β* are involved in the etiology of several diseases [17, 18]. Therefore, inhibition of pro-inflammatory cytokines is a strategy for prevention of immunological damage to organs [19]. Brennan et al. [20] have also reported enhanced renal expression of TNF-*α* and IL-1*β* in a SLE-prone murine model and that either TNF-*α* or IL-1*β* accelerated renal injury. Thus, it has been suggested that targeting the pro-inflammatory cytokines, such as TNF-*α* and IL-1*β*, is a desirable strategy for treatment of human SLE [21]. In this study, antroquinonol, the major active component of ACE, inhibited the production of TNF-*α* and IL-1*β* in LPS-induced RAW 264.7 cells, suggesting that this anti-inflammatory activity may contribute to the function of ACE in attenuation of the progression of lupus nephritis.

In conclusion, ACE reduced urine protein and creatinine levels and caused a reduction in the kidney glomerular basement membrane thickness, suggesting that ACE is able to protect the kidneys from the immunological damage characteristic of this autoimmune disease.

## Funding

Golden Biotechnology Corp., Taiwan.

## Figures and Tables

**Figure 1:** ACE maintains kidney function in SLE-prone mice. The NZB/W F1 mice were treated with different dosages of ACE (100, 200 and 400 mg kg^−1^) and prednisolone (1.25 mg kg^−1^) consecutively for 5 days per week for 12 weeks. At the end of experiment, blood of experimental animals was collected and serum was determined for the concentration of (a) serum BUN and (b) serum creatinine. Before the sacrifice of animals, urine was collected and then (c) urine protein and (d) urine creatinine were determined as described in Methods section.

**Figure 2:** ACE inhibits immunological kidney damage in SLE-prone mice. The NZB/W F1 mice were treated with different dosages of ACE (100, 200 and 400 mg kg^−1^) and prednisolone (1.25 mg kg^−1^) consecutively for 5 days per week for 12 weeks. At the end of experiment, blood of experimental animals was collected and serum was tested for anti-dsDNA IgG using a mouse anti-ds DNA IgG ELISA kit.

**Figure 3:** ACE inhibits glomerular basement membrane thickening in SLE-prone mice. The NZB/W F1 mice were treated with different dosages of ACE (100, 200 and 400 mg kg^−1^) and prednisolone (1.25 mg kg^−1^) consecutively for 5 days per week for 12 weeks. At the end of experiment, kidney was excised after sacrifice of animals and subject to pathological examination. The thickness of kidney glomerular basement membrane was determined by staining with PAS. The thickness was measured using a microscope.

**Figure 4:** Antroquinonol inhibits cytokine secretion in LPS-treated RAW 264.7 cells. The Raw 264.7 cells were treated with different concentrations of antroquinonol in the presence of LPS for 24 hours. The conditioned medium was subject to the determination of (a) TNF-*α* and (b) IL-1*β* levels. Data point of experiment was performed in triplicate and normalized by the induction of LPS as percentage. *P < .05, **P < .01, ***P < .001 versus LPS control, significant difference tested using student's *t*-test.

**Table 1:** Analysis of SLE indicators among SLE-prone NZB/W F1 mice.

Treatment (dose)	Body weight	Anti-dsDNA IgG	Urine protein	Urine creatinine
	(g) ^(a)^	(mg dL^−1^) ^(a)^	(mg dL^−1^) ^(a)^	(mg dL^−1^) ^(a)^
Control-ddH_2_O (10 mL kg^−1^)	35.4 ± 3.5	3.56 ± 2.79	89.2 ± 23.7	39.8 ± 12.5
Prednisolone (1.25 mg kg^−1^)	34.4 ± 3.9	4.07 ± 4.14	88.2 ± 14.6	38.0 ± 7.0
ACE (100 mg kg^−1^)	35.4 ± 3.6	4.86 ± 7.88	88.6 ± 16.7	33.7 ± 10.1
ACE (200 mg kg^−1^)	36.8 ± 2.8	5.06 ± 7.87	83.3 ± 20.2	34.6 ± 9.5
ACE (400 mg kg^−1^)	35.6 ± 4.6	5.29 ± 8.57	90.6 ± 19.8	40.6 ± 10.8
Normal (C57BL/6j mice)	18.2 ± 1.0	1.73 ± 0.53	75.1 ± 36.0	33.7 ± 15.7

^(a)^Data are expressed as mean ± SD.

**Table 2:** Body weight change in NZB/W F1 mice with treatment time ^(a)^.

Treatment (dose)	Week 0 ^(b),(c)^	Week 2 ^(b),(c)^	Week 4 ^(b),(c)^	Week 6 ^(b),(c)^	Week 8 ^(b),(c)^	Week 10 ^(b),(c)^	Week 12 ^(b),(c)^
Control-ddH_2_O	35.4 ± 3.5 (0%)	36.4 ± 4.0 (2.8%)	37.4 ± 3.2 (5.6%)	38.3 ± 3.9 (8.2%)	38.9 ± 4.1 (9.9%)	37.6 ± 3.6 (6.2%)	35.8 ± 4.9 (1.1%)
(10 mL kg^−1^)							
Prednisolone	34.4 ± 3.9 (0%)	34.0 ± 3.9 (−1.2%)	36.1 ± 4.0 (4.9%)	36.2 ± 4.2 (5.2%)	37.6 ± 3.5 (9.3%)	36.1 ± 3.3 (4.9%)	36.3 ± 3.4 (5.5%)
(1.25 mg kg^−1^)							
ACE	35.4 ± 3.6 (0%)	35.2 ± 3.3 (−0.6%)	36.7 ± 3.2 (3.7%)	36.7 ± 4.2 (3.7%)	37.1 ± 5.7 (4.8%)	37.8 ± 1.8 (6.8%)	36.5 ± 3.1 (3.1%)
(100 mg kg^−1^)							
ACE	36.8 ± 2.8 (0%)	37.4 ± 2.6 (1.6%)	37.5 ± 3.0 (1.9%)	38.3 ± 3.6 (4.1%)	38.7 ± 4.9 (5.2%)	38.9 ± 2.1 (5.7%)	39.0 ± 2.0 (6.0%)
(200 mg kg^−1^)							
ACE	35.6 ± 4.6 (0%)	35.5 ± 4.5 (0%)	36.7 ± 4.5 (3.1%)	36.8 ± 5.0 (3.4%)	37.2 ± 6.1 (4.5%)	37.0 ± 8.2 (3.9%)	37.9 ± 6.3 (6.5%)
(400 mg kg^−1^)							

^(a)^Fifty NZB/W F1 female mice were divided into 5 groups of 10 each. Different doses of ACE and prednisolone were administrated by gavages for 5 consecutive days per week for 12 weeks.

^(b)^Data are expressed as mean ± SD.

^(c)^Values in parentheses indicate percent increase in body weight compared to initial body weight.
